# Contemporary Concepts in Osseointegration of Dental Implants: A Review

**DOI:** 10.1155/2022/6170452

**Published:** 2022-06-14

**Authors:** Chandrashekhar Pandey, Dinesh Rokaya, Bishwa Prakash Bhattarai

**Affiliations:** ^1^Master Degree Student in Oral and Maxillofacial Surgery (International Program), Walailak University International College of Dentistry, Walailak University, 87 Ranong 2 Road, Nakhon Chai Si, Dusit, Bangkok 10300, Thailand; ^2^Department of Clinical Dentistry, Walailak University International College of Dentistry, Walailak University, 87 Ranong 2 Road, Nakhon Chai Si, Dusit, Bangkok 10300, Thailand

## Abstract

In a society highly conscious of esthetics, prosthetic rehabilitation of lost teeth with tissue-integrated implants has gained wide acceptance and demand by patients and clinicians. The backbone of these tissue-integrated implants is the biotechnical process of osseointegration. Although the concept has been introduced and discussed for ages, the deepening knowledge about its cellular and molecular mechanisms has led the researchers to borrow further into the factors influencing the process of osseointegration. This has aided in the hastening and improving the process of osseointegration by exploiting several, even the minutest, details and events taking place in this natural process. Recently, due to the high esthetic expectations of the patients, the implants are being loaded immediately, which demands a high degree of implant stability. Implant stability, especially secondary stability, largely depends on bone formation and integration of implants to the osseous tissues. Various factors that influence the rate and success of osseointegration can either be categorized as those related to implant characteristics like the physical and chemical macro- and microdesign of implants or the bone characteristics like the amount and quality of bone and the local and systemic host conditions, or the time or protocol followed for the functional loading of the dental implant. To address the shortcomings in osseointegration due to any of the factors, it is mandatory that continuous and reliable monitoring of the status of osseointegration is done. This review attempts to encompass the mechanisms, factors affecting, and methods to assess osseointegration, followed by a discussion on the recent advances and future perspectives in dental implantology to enhance the process of osseointegration. The review was aimed at igniting the inquisitive minds to usher further the development of technology that enhances osseointegration.

## 1. Introduction

In a society too conscious about esthetics and appearance, it is a must that the teeth, one of the major attributes of the smile, be healthy and long-lived. However, the teeth cannot be restored several times and are lost for various reasons. Apart from compromising esthetics, tooth loss has vivid and enormous consequences on the local and general health of the patient. Modern dentistry aims to restore the oral health of patients in a predictable fashion. Depending on an individual's local, environmental, physiological, mental, and financial status, the lost teeth are replaced with the best possible alternative.

Osseointegration, a concept introduced by Per-Ingvar Branemark, widened the room for restorative options for partially and completely edentulous patients. The idea exploits the clinical usage of biotechnology and continues to be a boon for dental patients and clinicians.

Since then, several attempts have been made to aptly define the concept of osseointegration. Branemark initially defined osseointegration as “a direct structural and functional connection between ordered living bone and the surface of a load-carrying endosseous implant at the light microscopic level” [1]. Next, the American Academy of Implant Dentistry (1986) defined it as “contact established without the interposition of nonbone tissue between normal remodeled bone and an implant, entailing a sustained transfer and distribution of load from the implant to and within the bone tissue” [2]. Later, the glossary of prosthodontic terms-8 (GPT-8) defined it as “the apparent direct attachment or connection of osseous tissue to an inert, alloplastic material without intervening connective tissue” [3].

However, these age-old descriptions fail to consider a vital parameter of the newly formed osseous tissue, i.e., the quality of bone. Therefore, the definition of osseointegration must thoroughly blend several other parameters as well, such as prosthetic stability under functional loads, apposition of new bone without the interposition of connective tissue, lack of mobility of implant in relation to the surrounding tissue under functional loading, and normal bone and marrow tissues evident on the implant surface at the light and electron microscopic levels [4].

This review was aimed at including facts on dental implant osseointegration outlined in the contemporary literature. To identify pertinent articles on osseointegration of dental implants, we conducted a literature search on PubMed, PubMed Central, and Medline using keywords like “osseointegration,” “implant stability,” “bone-to-implant contact,” and “bone-to-implant interface.” The search yielded a total of 1,080 articles, which were scrutinized to gather relevant information for this review.

## 2. Historical Background

At the Lund and Goteborg universities, the concept of osseointegration has been under extensive research since 1952. The concept stemmed from the microscopic studies on rabbit fibula bone marrow, uncovered with gentle surgery and inspected at high resolution under a modified intravital microscope [1].

In the early 1960s, studies evaluated the reaction of bone marrow and joint tissue to mechanical, chemical, thermal, and rheologic tissue injury. With the possibility of osseointegration being evident in most studies, Branemark, in one of the studies reviewing microcirculation, observed bone tissue growing into narrow spaces in titanium and the titanium chambers that got incorporated in the bone tissue inseparably [1].

Due to the lack of methods enabling intact bone to metal specimens, histological evidence remained inadequate and secondary until the early 1970s. Then, in the mid-1970s, it was for the first time that Schroeder histologically demonstrated the evidence of osseointegration and successfully proved a direct bone-to-implant contact [5, 6]. Later, Cameron et al. [7] in 1973 suggested that bone grows on a biocompatible material only when the movement of both the bone and the implant is restricted.

## 3. Expanding the Understanding of Osseointegration

### 3.1. The Cellular and Molecular Physiology of Osseointegration

A physiological event during the integration of bone and implant follows the process of primary bone healing. First, the implant is placed in the bone, and water forms a layer in the surrounding within nanoseconds, facilitating the absorption of protein and other essential molecules [8]. Then, within the next 30 seconds to several hours, intercellular matrix proteins derived initially from the interstitial fluid and blood and later from the cellular activity coat the implant surface with a structure, composition, and inclination dictated by the surface type [9]. Via this protein layer, cell adhesion, migration, and differentiation are initiated, helping an interaction of the cells with the implant surface for several hours or days [10]. Further adjustments are introduced by the extracellular matrix proteins (ECM), cytoskeletal proteins, the cell surface-binding proteins and the binding topography, and the chemical characteristics and ion release [11]. The ECM proteins transmit decodable data to the cells and the cohesive structures, determining the shape, mobility, polarity, gene expression, survival, and proliferation of cells [12–14]. This data transmission occurs in various proteins like collagen I, fibronectin, osteopontin, osteonectin, osteoadrin, bone sialoprotein, and specific plasma proteins like *α*2HS glycoprotein sufficing the needs as cell adhesion interfaces and messengers for the cell to cell or cell to protein interactions [9]. Chronological cellular and molecular events leading to osseointegration after implant placement have been concluded in Table 1.

The cellular and molecular events of osseointegration are shown in Figures 1–3.

When titanium is exposed to air, a thin layer of titanium oxide forms on the surface, protecting the highly reactive titanium surface from biological attack while improving the wear resistance. However, the layer also influences biomineralization by letting the Ca^2+^ and PO_4_^3-^ adsorb on the surface [22, 23]. Once activated, osseointegration follows the common biological events subdivided into three stages: the stage of implant incorporation in the bone by the formation of woven bone, the stage of bone mass adaptation (lamellar and parallel-fibered bone) to the load, and finally the stage bone structure adaptation (bone remodeling) to the load.

### 3.2. Osseointegration versus Fracture Healing

Although the process of osseointegration has been rounded off to be similar to that of fracture healing, where the lamellar bone replaces the initial formed woven bone, the progenitor cells at the site of osseointegration, unlike those at the site of fracture healing, entirely differentiate into osteoblasts followed by intramembranous ossification, with no population of cells being differentiated into chondroblasts and aiding in endochondral ossification [4]. Another major difference lies in the presence or absence of an implant and implant surface. Unlike in fracture sites, a major part of the bone gap is filled with the body of the implant, minimizing the area to be refilled by new bone. Moreover, the surface properties of the implant and the novel surface treatments further incite an osteogenic cell response [24].

## 4. Requisites for Successful Osseointegration

Successful osseointegration depends on the interrelationship of various confounding factors such as the biocompatibility of the material of implant, the macro- and microscopic topography of implant surface, design of the implant, bone morphology and quality at the implant site, the surgical technique employed, stability of local and systemic health during the healing phase, and the loading conditions and protocol followed [25–28]. The greatest challenge for clinicians in obtaining successful osseointegration is that all these factors must be controlled simultaneously.

### 4.1. Factors Determining the Success and Failure of Osseointegration

For a successfully long-lived endosseous implant, the complex process of osseointegration needs to be thoroughly kept in check by controlling the various influential factors.

#### 4.1.1. Implant Characteristics

*Geometry of Implant:* the growth of the bone occurs preferentially on the elevated or the protruded extensions on an implant surface, such as the ridges, crests, and edges of threads. Moreover, the shape of the implant is also an essential determinant as it governs the surface area available for the transfer of stresses and the primary implant stability. A threaded implant offers greater functional surface area than the smooth-sided cylindrical or tapering implants, as it can be rigidly fixated, thereby limiting the microenvironment during wound healing. Smooth-sided implants need an additional surface treatment, and the taper, when incorporated, reduces the surface area available for osseointegration [29]. Studies have shown that implant design with grooves oriented +60° (downwards) to the long axis of the implant attracts higher densities of osteocytes in the peri-implant area [30].

*Width and Length of Implant*: the greater the dimensions of an implant, the greater is the surface area provided for osseointegration. However, increasing the length beyond a limit must be avoided as it may not allow the proportionate transfer of forces [29].

*Microdesign of Implant:* surface modification of implants is performed to achieve a biocompatible and bioactive surface. Commercially, pure titanium has been the standard material for endosseous implants. It is highly reactive and forms a passivation layer of titanium oxides compatible with the tissues without becoming incorporated. Furthermore, treatments like sandblasting with aluminum oxide or titanium oxide have been shown to permit better adhesion, proliferation, and differentiation of osteoblasts [31]. Likewise, titanium plasma-sprayed surface increases the area of the bone-implant interface to as high as 600%, stimulating osteogenesis. A recent dual acid-etched technique yields a higher adhesion of platelet genes and the expression of extracellular genes. The newly introduced technique of combining the advantages of sandblasting and acid-etching, known as the sandblasted, large-grit, acid-etch (SLA) implant surface, exhibits greater alkaline phosphatase activity in osteoblast-like cells than other techniques [32]. Apart from these techniques, other surface treatments like anodization of surface, laser treatment, and tricalcium phosphate coatings have also been tried. The tricalcium phosphate coatings have osteoinductive properties acting as scaffolds or nidus for bone growth.

Moreover, by such coating of the implant surface, the yielded bioreactive bond with the bone and the physical interlocking enhances osseointegration [33]. Likewise, hydroxyapatite coatings exhibit similar properties that increase the functional surface area, and the bone-to-implant interface is greater than that achieved by any former surface treatments. The hydroxyapatite surfaces are conducive to the morphogenic activities of osteogenic cells, along with providing an accelerated interfacial bone formation and maturation [34]. Furthermore, to shorten the recovery period and aid in early functional loading that generally hampers the process of osseointegration, a capacitively coupled electric field is used to stimulate early and rapid osteogenesis by stimulating the pluripotent mesenchymal cells [35]. Likewise, to shorten the time lapse between extraction of tooth and implant osseointegration, bovine osteogenic protein insertion into unmodified sockets with implants has been tried with positive results [36].

#### 4.1.2. Bone Characteristics

The bone is the bed in which the implant is placed, and its health is one of the most crucial determining factors in osseointegration. A bone that has been irradiated or has suffered from osteoporosis poses undesirable hurdles during osseointegration. Thus, it is advocated that some delay should be allowed after irradiation to place an implant, or the healing conditions are improved with hyperbaric oxygen therapy. Other host bone deterrent factors include smoking history or systemic conditions like diabetes mellitus or hypertension. Moreover, ridge augmentation or bone grafting must be done to address resorbed or insufficient volume of alveolar ridges to allow sufficient osseointegration.

#### 4.1.3. Intraoperative Factors

Restricting the tissue damage to minimal and maintaining temperatures of bone below the hazardous levels with low-speed surgical drilling are essential to avoid inadvertent bone necrosis. For example, a temperature of 47°C for 1 min initiates bone tissue necrosis.

#### 4.1.4. . Implant Loading

Sufficient osseointegration is achievable with a thoroughly established primary implant stability. Over the years, various implant loading protocols have been followed with variable clinical outcomes. Esposito et al. conducted a systematic review of randomized control trials to assess the effect of immediate occlusal loading during the bone healing phase. Still, the authors chose not to say whether avoiding occlusal contacts during the osseointegration phase was beneficial [37]. Similarly, in a systematic review and meta-analysis by Chen et al. [38] comparing the efficacy of immediate versus conventional implant loading, the authors concluded that immediate loading could achieve comparable implant survival rates compared to early loading, but not when compared to conventional loading. Donati et al. [39] compared the osseointegration of immediate functionally loaded implants and nonloaded implants histologically in terms of bone-to-implant contact percentage and bone quality formed in the peri-implant region. The percentage of bone to implant contact was not significantly different; additionally, the newly formed peri-implant bone in the immediate functionally loaded implants was significantly thicker.

## 5. Assessment of Osseointegration

Continuous and reliable monitoring of the status of osseointegration is recommended for the success of implants. Implant stability, more specifically the secondary implant stability, reflects the quality of osseointegration. Microscopic or histological analysis has been the standard methodology for assessing osseointegration status for centuries; however, due to its invasiveness, other methods such as radiographic, cutting torque resistance, reverse torque, and model analyses are now being used.

### 5.1. Histomorphometric Assessment

Histological assessment provides an in-depth knowledge of the bone quality around the implant, contact percentage between bone and implant, type of bone formed, and morphological characteristics of the osteocytes, such as size, orientation, and alignment to the bone lamellae, number and density, proximation to blood vessels, and lacuno-canalicular interconnectivity between neighboring and distant osteocytes. However, due to the invasiveness of the analysis, it is reserved for nonclinical studies or experiments [40, 41].

### 5.2. Radiographic Assessment

Radiographic visualization through the routinely used techniques is a noninvasive way to assess osseointegration. Chopra et al. evaluated osseointegration using a digital orthopantomogram and cone-beam computed tomography (CBCT). The osseointegration was found to be 0.03 mm at the apical portion of implants and 0.04 mm at the crestal bone height on digital orthopantomogram and 0.01 mm at the apical portion on CBCT after three months of implant placement. They suggested that both orthopantomogram and CBCT are efficient at assessing osseointegration. Although computed tomography lures a clinician as a better technique for evaluating the same, one must restrict its use to the point of benefit with the lowest radiation doses [42]. It is essential to differentiate between the bone formed by contact and distant osteogenesis. At times, failure may occur due to poor bone-to-implant contact despite large amounts of bone in the implant threads. This differentiation is difficult on routine radiographs, and in fact, even the highly sophisticated ex vivo X-ray microcomputed tomography cannot resolve the first few millimeters around the implant surface [43]. Jung et al. [44] tested the use of synchrotron radiation X-ray microimaging to evaluate osseointegration. They used unmonochromatic synchrotron radiation to study the bone-to-implant interface and compared the yielded image quality with microcomputed tomography images and conventional dental radiographs, focusing the evaluation mainly on the osseous contact at the bone-to-implant interfaces. They unveiled that the synchrotron radiation imaging technique provided finer details of the osseous contact. Thus, they expected this technique to bring an enormously positive influence on the studies on the evaluation of osseointegration.

### 5.3. Clinical Assessment

The tests used in clinical practice are either invasive or noninvasive. The tensional test, which involves detaching the implant plate from the supporting bone, was one of the invasive tests used in the past. Later, Branemark tested osseointegration by applying lateral load to the implant fixture [45]. Similarly, the push- or pull-out test, which assesses strength and stiffness at the bone-implant interface by applying a load parallel to the interface, is only applicable to nonthreaded cylindrical implants and is technique dependent. The reverse torque test, proposed by Roberts et al. [46] and later developed by Johansson and Alberktsson to assess secondary stability, may rotate the implants and destroy the bone-implant interface when torque is applied. Furthermore, due to varying threshold limits among patients, implant material, and bone quality and quantity, the test cannot quantify the degree of osseointegration [25].

Recently, the focus has shifted to noninvasive methods that now outnumber the invasive ones. These noninvasive methods can be enlisted from the simplest one, involving the perception of a surgeon acquired by the cutting resistance and seating torque during implant placement. However, this typically measures the primary stability of the implant, not reflecting the real picture of osseointegration at the healing stages. Similarly, insertion torque values can be used to assess the quality of bone in various parts of the jaw during implant placement, but they cannot evaluate the secondary stability provided by the new peri-implant bone formation and remodeling [47]. A simpler test, the percussion test using a metallic instrument, based upon the science of vibration, acoustics, and impact response, can evaluate osseointegration, with the “crystal-like” clear sound indicative of successful osseointegration and a dull sound expressive of otherwise. However, it is a subjective method and cannot be standardized [48]. Kaneko et al. [49] introduced an advanced technique using the forced excitation of steady-state waves that helped examine the mechanical vibrations at the bone-implant interface displayed on an oscilloscope screen. A similar approach, the resonance frequency analysis, suggested by Meredith, measures bone densities at different time points using vibrations and the principle of structural analysis. The implant is shattered at a constant amplitude by an amplifier vibrated by a sinusoidal signal (5-15 kHz). A high-frequency resonance indicates a strong bone-implant interface. This method has been widely used to assess osseointegration in clinical settings. The Osstell (electronic technology resonance frequency analysis) and Osstell mentor are advanced versions of this technique (magnetic technology resonance frequency analysis) [50].

## 6. Recent Approaches and Future Perspectives in Implant Technology to Enhance Osseointegration

### 6.1. Macrotopography Enhancements

Since the implant surface topography is a determinant of cell adhesion and osteoblast differentiation required for osseointegration, the diameter of the inner thread of an implant must be equal to the dimensions of the socket, helping achieve high primary stability by friction. The outer thread diameter should be the same as the implant cavity diameter, allowing granulation tissue formation and subsequent osseointegration. Additionally, the instrumentation should be between the inner and outer threads, aiding bone remodeling induced by compression and healing chambers required for the migration of osteogenic cells [51–53].

### 6.2. Microtopography Enhancements

Microtopography is linked to microroughness, aiding the attachment of osteogenic cells and bone deposition in the range of 1-100 *μ*m and can be enhanced with several manufacturing techniques, as listed in Table 2.

### 6.3. Nanotopography Enhancements

While microtopography acts at the cellular level of osseointegration, nanotopography is supposed to act at an additional protein level. It exerts effects through physical, chemical, and biological routes, increasing the adhesion of osteogenic cells and promoting osseointegration. Some of the recently introduced methods are enlisted in Table 3.

### 6.4. Surface Wettability Improvements

Improving the wettability (making the surfaces as hydrophilic as possible) avoids denaturation of proteins and has a higher affinity for cell binding domains, improving cellular attachments. This also accelerates osseointegration by promoting the differentiation and maturation of osteoblasts [69].

### 6.5. Photofunctionalization

Implant surfaces treated with UV radiation have enhanced bioactivity and osseointegration potential due to alteration of the titanium dioxide surface layer. Furthermore, UV light enhances osteoconductivity by promoting cell and protein interactions with the implant surface. Also, it reduces surface hydrocarbon, improves wettability, increases protein adsorption and cellular attachment to titanium surfaces, and restores bioactivity that gets diminished due to age-related degradations [70].

### 6.6. Surface Coatings

Implant surfaces coated with growth factors (e.g., platelet-derived growth factors, transforming growth factor-beta, fibroblast growth factor, vascular endothelial growth factor, and bone morphogenetic proteins), extracellular matrix proteins, peptides, and messenger molecules like sclerostin hasten the process of osseointegration, being the natural players in the process. Furthermore, the surfaces are being coated with drugs like bisphosphonates to combat any limiting local or systemic host conditions [71].

### 6.7. Local Drug Delivery

According to a study conducted by Rostom and Faroukabdulla, local melatonin administration increases bone density, improving the process of osseointegration around immediately loaded implants [72].

## 7. Recent Advances in Dental Implant Biomaterials

Metals and their alloys are long being used as implant materials in human body largely due to their properties of biocompatibility and acceptable physical and chemical properties. When it comes to dental implants, titanium and titanium alloys have been the biomaterials of choice [73]. Ceramic-based materials (e.g., zirconia, zirconia toughened alumina, and alumina toughened zirconia) are also gaining popularity as the biomaterials for dental implants. Zirconia has better flexural strength, higher fracture resistance, and releases lesser ions compared to titanium. Additionally, the zirconia implants have better osseointegration and esthetic properties compared to titanium implants [74].

Tantalum is another metal that is currently being studied as a biomaterial for dental implants. Porous tantalum has greater resistance against corrosion and has been used with success as implant material in orthopedic surgeries for improving angiogenesis and wound healing [75]. Studies on the use of tantalum as a dental implant biomaterial are few. In their in vitro study, Piglioncio et al. concluded that porous tantalum has greater osseointegration capacity than the currently available smooth or roughened titanium implants [76]. In another retrospective study by Edelmann et al., the porous tantalum trabecular metal-enhanced titanium implants showed significantly less peri-implant bone loss compared to the regular titanium implants [77].

Polyetheretherketone (PEEK) is an organic polymer that has been gaining popularity as a biomaterial for dental implants and prosthesis. The higher modulus of elasticity of PEEK compared to titanium allows it to dissipate masticatory forces evenly when used as a dental implant. Moreover, PEEK also possesses superior color stability and higher abrasion resistance than zirconia [78]. However, without any surface modifications, PEEK does not produce osseointegration; only mechanical interlockings are formed at the PEEK-bone interface. Therefore, to enhance osseointegration, surface modifications are done with hydroxyapatite, titanium oxide, and magnesium phosphate sprays. Mishra and Chowdhary in their systematic review on PEEK as a potential alternative to titanium dental implant concluded that upon surface modification, PEEK showed improved cell adhesion, proliferation, and osseointegration [79]. Nevertheless, more clinical trials are required to establish PEEK as the replacement for titanium as dental implant biomaterial.

## 8. Surgical Techniques to Enhance Dental Implant Osseointegration

One of the factors that influences successful osseointegration is the primary stability of the dental implant while insertion. In recent years, undersized drilling has been advocated to achieve sufficient insertion torque especially in regions of the jaws where the alveolar bone has lesser density. In the undersized drilling, the final drill is of lesser diameter than the fixture diameter, which allows the lateral compression of the bone during the fixture installation. This enables the fixture to achieve higher primary stability. The effectiveness of the undersized drill to achieve higher primary stability has been shown in an experimental study by Tobassum et al. [80] and in a systematic review by Stocchero et al. [81].

Another surgical technique that improves osseointegration by improving the primary stability of the dental implant is the osteotome technique. This technique basically involves the sequential expansion-condensation of the alveolar bone using successive osteotomes of greater diameter. The technique is believed to reduce the microdeformations and maximize the preservation of remaining bone [82]. The osteotome technique is suggested to be an effective method to gain higher primary implant stability than the conventional drilling technique especially in low density alveolar bone [83, 84].

Osseodensification is one of the contemporary drilling techniques aimed at bone preservation and compaction during the preparation of implant bed. This technique helps to gain high initial primary stability than the conventional drilling ultimately resulting in higher degree of osseointegration. Unlike conventional drilling which removes the bone from the osteotomy walls, osseodensification is a nonsubtractive technique that condenses the bone chips removed during the drilling on the osteotomy walls. As a result, a compact layer of autogenous bone is created around the implant surface after insertion [85]. Inchingolo et al. have done a systematic review and meta-analysis comparing insertion torque, bone to implant contact, and bone area fraction occupied between osseodensification and conventional drilling. All of the parameters measured were higher for osseodensification compared to the conventional drilling, which suggests that osseodensification is a superior technique to achieve better osseointegration especially in areas of low bone density [86]. However, the results on osseodensification are primarily from animal studies; hence, clinical trials in human are warranted to confirm those results.

## 9. Conclusion

A successful replacement of the natural tooth with the help of tissue integrated implants is solely based on successful osseointegration. Therefore, an adequate understanding of the process of osseointegration, its prerequisites, and factors promoting and limiting osseointegration has been helping and shall help enormously in the near future to exploit every related parameter and improve and hasten the process of osseointegration.

## Figures and Tables

**Figure 1:** Day 1 and day 2 after implant placement. Day 1: secretion of growth factors and migration of undifferentiated osteoblasts and pluripotent stem cells towards implant surface. Day 2: local ischemia and necrosis followed by recruitment of neutrophils and macrophages.

**Figure 2:** Day 3 and day 4 after implant placement. Day 3: activation of osteoblast-related transcription factors by the cells around the implant. Day 4: resorption of necrotic bone and deposition of new bone at the bone-implant interface.

**Figure 3:** Day 28 and 12th week after implant placement. Day 28: formation of new layer of bone adjacent to implant through contact and distant osteogenesis. End of 12th week: formation of a mature lamellar bone connection with the titanium surface.

**Table 1:** Chronology of cellular and molecular events of osseointegration after implant placement.

Timeline after implant placement	Cellular/molecular event
1^st^ day	(i) Secretion of growth factors by water molecules and platelet absorption at the site of implant placed [15] (ii) Nondifferentiated osteoblasts stick to the implant surface through the aid of fibronectin [16] (iii) Migration of pluripotent mesenchymal cells along the implant surface, with their function dependent on the local oxygen tension and regulatory growth factors, which are further dependent on the position of implant and angiogenesis [17, 18]
2^nd^day	(i) Local ischemia and necrosis toward the center of the implant site due to the capillary breakdown [19] (ii) Neutrophils become the predominant cells, followed by macrophages becoming dominant, forming clots and tissue necrosis
3^rd^ day	(i) Activation of Runx2 and Op (osteoblast-related transcription factors) by the cells around the implant [4]
4^th^ day	(i) Necrotic bone resorption and the formation of some bone-implant interface [20]
5^th^ day	(i) Evidence of new bone formation and initiation of mineralization and matrix remodeling as indicated by the alkaline phosphatase activity [4]
7^th^ day	(i) Recognizable bone matrix cohesion on surface of implant [4] (ii) Bone-to-implant contact attained is 35.8% [21]
16^th^ day	(i) Implant surface becomes entirely coated with mineralized tissues, osteoid, and dense matrix [20]
28^th^ day	(i) Complete binding of bone along the implant surface formation of a volume of tissue layer comprised of collagen fibers and osteoblasts adjacent to the implants; alignment of collagen fibers running parallel to the implant's surface. Bone-to-implant contact of 46.3% is reached [21] (ii) Bone regeneration: (i) *Contact osteogenesis*: from implant surface towards the bone (30% faster shaping of bone); as a response to the implant surface's physicochemical properties [9, 19] (ii) *Distant osteogenesis*: from the margin of bone to the surface of the implant; de nova formed bone is of woven type [9, 19]
End of the 12^th^ week	(i) Establishment of a mature lamellar bone connection with the titanium surface leading to uniformity of bone formed on the implant's surface [20]

**Table 2:** Outcomes of microtopography enhancement techniques.

Technique	Rationale	Preclinical data	Clinical data
Sandblasting and acid-etching	Sandblasting and acid-etching increases microroughness and surface area	Superior bone-to-implant contact (50-60%) at 3 and 6 months as compared to plasma-spraying (30-40%) and electropolished (20-25%) implants [54]. Superior bone anchorage with higher removal torque values in minipig models [55].	Implant survival rate: 95.1%-98.8% [56, 57]
Grit-blasted, acid-etched, and neutralized implants	Macroroughness by grit-blasting; hydrophobic surface is changed to hydrophilic, increasing the wettability (water contact angle 0^o^) [58]	Even the immediately loaded implants showed a higher degree of bone formation and satisfactory bone-to-implant contact [59, 60]	Success rate after one year of implant placement was 99.6% [61]

**Table 3:** Outcomes of nanotopography enhancement techniques.

Technique	Rationale	Preclinical data	Clinical data
Discrete crystalline deposition	CaP particles (20-100 nm) deposited on a double acid-etched surface by a sol-gel process exert a high adhesive force on the implant surface; bacterial adhesion is reduced [62, 63]	Disruption force required at the bone-implant interface is high; high osteoconduction [64]	One year survival rate 94.9%-99.4% [65, 66]
Laser ablation	Generates a pattern of nanoscale microchannels that act as a biological seal by eliciting the connective tissue and bone attachment, inhibiting epithelial down growth [67]	Dense cervical seal prevents apical migration of junctional epithelium [67]	Two-year survival rate 96.1%; long-term comparative results not yet available [68]
